# Anticancer activity of 2’-hydroxyflavanone towards lung cancer

**DOI:** 10.18632/oncotarget.26329

**Published:** 2018-11-16

**Authors:** Sanjay Awasthi, Sharad S. Singhal, Jyotsana Singhal, Lokesh Nagaprashantha, Hongzhi Li, Yate-Ching Yuan, Zheng Liu, David Berz, Henry Igid, William C. Green, Lukman Tijani, Vijay Tonk, Aditya Rajan, Yogesh Awasthi, Sharda P. Singh

**Affiliations:** ^1^ Division of Hematology and Oncology, Department of Internal Medicine, Texas Tech Health Sciences Center, Lubbock, TX 79430, USA; ^2^ Department of Medical Oncology, Beckman Research Institute, City of Hope National Medical Center, Duarte, CA 91010, USA; ^3^ Bioinformatics Core Facility, City of Hope National Medical Center, Duarte, CA 91010, USA; ^4^ Beverly Hills Cancer Center, Los Angeles, CA 90211, USA; ^5^ Department of Pediatrics, Texas Tech Health Sciences Center, Lubbock, TX 79430, USA; ^6^ Department of Biochemistry and Molecular Biology, the University of Texas Medical Branch, Galveston, TX 77555, USA

**Keywords:** 2’-hydroxyflavanone, lung cancer, small cell lung cancer, non-small cell lung cancer, Ralbp1

## Abstract

In previous studies, we found that 2'-hydroxyflavonone (2HF), a citrus flavonoid, inhibits the growth of renal cell carcinoma in a VHL-dependent manner. This was associated with the inhibition of glutathione S-transferases (GSTs), the first step enzyme of the mercapturic acid pathway that catalyzes formation of glutathione-electrophile conjugates (GS-E). We studied 2HF in small cell (SCLC) and non-small cell (NSCLC) lung cancer cell lines for sensitivity to 2HF antineoplastic activity and to determine the role of the GS-E transporter Rlip (Ral-interacting protein; RLIP76; RALBP1) in the mechanism of action of 2HF. Our results show that 2HF induced apoptosis in both histological types of lung cancer and inhibited proliferation and growth through suppression of CDK4, CCNB1, PIK3CA, AKT and RPS6KB1 (P70S6K) signaling. Increased E-cadherin and reduced fibronectin and vimentin indicated inhibition of epithelial-mesenchymal transition. Additionally, 2HF inhibited efflux of doxorubicin and increased its accumulation in the cells, but did not add to the transport inhibitory effect of anti-Rlip antibodies alone. Binding of Rlip to 2HF was evident from successful purification of Rlip by 2HF affinity chromatography. Consistent with increased drug accumulation, combined treatment with 1-chloro-2, 4-dinitrobenzene, reduced the GI_50_ of 2HF by an order of magnitude. Results of *in-vivo* nude mouse xenograft studies of SCLC and NSCLC, which showed that orally administered 2HF inhibited growth of both histological types of lung cancer, confirmed *in-vitro* study results. Our result suggest that Rlip inhibition is likely a mechanism of action. Our findings are basis of proposing 2HF as therapeutic or preventative drug for lung cancer.

## INTRODUCTION

Lung cancer is the most frequently diagnosed cancer and the leading cause of cancer death worldwide, the most common cancer diagnosed in men with more than 1.5 million persons annually [1, 2]. These numbers are a stark reminder of the inadequacy of present preventative and therapeutic interventions for this disease epidemic. Prevention of lung cancer is of utmost importance because treatment of lung cancer remains woefully inadequate and represents a massive social and financial burden on healthcare systems costing over $12 billion in the United States in 2010 alone [3]. Because smoking cessation strategies have yet proven insufficient, development of effective and inexpensive pharmacological means to prevent and treat lung cancer worldwide is needed. Preventative agents with therapeutic activity would be of particular importance since present systemic therapies for lung cancer including chemotherapy, targeted signaling inhibitors and novel immunotherapies fail to cure the vast majority of patients, and are plagued with obstacles including toxicity, narrow spectrum of activity, de-novo or acquired resistance and inordinate costs [4–7].

Increased risk of carcinogenesis, genetic instability, resistance to therapy, and poor survival outcomes are strongly linked to loss of normal functions of p53, a stress-responsive tumor suppressor protein (encoded by the human TP53 gene) that normally halts cell cycling and activates DNA repair mechanism in response to DNA damage caused by cigarette smoke genotoxins. TP53 is mutated in 94%, of small cell lung cancer (SCLC) [8], 94% of squamous (SqCA) [9], and 54% of adenocarcinoma (AdCA) [10] subtypes of non-small cell lung cancer (NSCLC). The former two types of lung cancer, i.e. SCLC and SqCA are mainly treated with chemotherapy while subsets of adenocarcinoma that have targetable oncogenic driver mutations such as EGFR, ROS1, or ALK rearrangements are treated with Tyrosine Kinase Inhibitors(TKIs) [11, 12]. Because TP53 also normally activates apoptosis of cells with irreparable genotoxic injury, its loss allows the survival of genetically damaged cells. As these damaged cells accumulate, they develop increasing genetic instability that accelerates carcinogenesis [13, 14]. In response to genotoxic stress, p53 also activates stress-responsive xenobiotic detoxification and drug efflux mechanisms that protect cells from acute injury through metabolic detoxification and removal of genotoxins. Long-term exposure to genotoxic stress in persons addicted to cigarettes eventually overwhelms these defenses because rapidly proliferating cells with genomic instability can eventually acquire critical DNA lesions that permit pre-cancerous cells to cross the threshold of malignant transformation. Though genoprotective xenobiotic defenses exert beneficial effects by reducing exposure to genotoxins on normal or pre-malignant cells, their anti-apoptotic activity also permits survival and accumulation of pre-malignant cells that harbor increasing numbers of cancer promoting DNA lesions. After malignant transformation, the cancer-protective effects of xenobiotic defenses actually become cancer promoting since their anti-apoptotic activities promote survival of cancer stem cells and mediate drug-resistance through anti-apoptotic, drug-metabolism, and drug-efflux processes.

Glutathione (GSH, γ-glutamyl-cysteinyl-glycine) is a sulfhydryl-containing tripeptide utilized by the mercapturic acid pathway (MPy) of GSH-mediated metabolism of genotoxic electrophilic xenobiotics (E) or reactive mutagens generated upon mono-oxygenation of xenobiotics by cytochromes P450. Glutathione S-transferases (GST) catalyze the next reaction, conjugation of GSH with electrophilic genotoxins (E) to form glutathione-electrophile thioether conjugates (GS-E) that are removed from cells through active transport by the down-stream GS-E transporters (the next step of MPy), and subsequently metabolized and excreted by the kidney as mercapturic acids [15–17]. Many phenolic antioxidants have been shown to exert protective effects against carcinogenic chemical in numerous experimental models of cancer. These antioxidants exert their cancer preventative activities though free radical scavenging and through activation of endogenous biological antioxidant enzyme and suppression of pro-inflammatory/pro-oxidant pathways such as NFκB. The cancer-preventative effect of antioxidant on augmenting endogenous genoprotective defenses characteristically include increased GST expression and decreased p450 expression. Indeed, this characteristic feature has proven to an excellent screen for identifying cancer-preventative antioxidants [18]. Despite success in short-lived animal models, phenolic antioxidants have not yet proven to be effective in preventives of lung cancer in humans [19]. The dual role of GSTs in cancers, ameliorating carcinogenic mutations but protecting mutated cells from undergoing apoptosis may be a reason for failure of many antioxidants in lung cancer prevention trials. The contrasting effect of stress-defense mechanisms on normal vs. transformed cells underlies a fundamental problem with phytochemical candidates for lung cancer prevention because their genoprotective effects are mediated by inducing biological antioxidant mechanisms, particularly glutathione-linked enzymes of the mercapturic acid pathway (MPy). In support of this model, the expression of GSTs is increased in lung cancer portends poor survival and resistance to chemotherapy as well as radiotherapy. Furthermore, GST inhibitors are in development as anticancer agents to modify treatment resistance and shortened survival associated with high GST expression in cancer patients [20]. All antioxidants are also oxidant at higher concentrations [21, 22], thus at high concentrations they can suppress GSTs; this would serve a therapeutic function. At low concentrations, however, they could reduce oxidative damage though GST induction and be cancer preventative. Because early lung cancers have previously not been readily detectable at an early curable stage, the effectiveness of low-dose antioxidants in lung cancer prevention could be underestimated by inclusion of patients with preclinical malignancy.

The U.S Preventive Services Task Force recently approved Lung Cancer Screening with low-dose CT for patients aged 55 to 88 who had a smoking habit of 30 pack-years or had quit within the past 15 years. The advent of effective CT-based lung cancer screening has resulted in increasingly frequent identification of very small (2–4 mm) lesions for which biopsies are not feasible, thus it is unclear whether an antioxidant would be best used as a primary preventative (low-dose) or secondary preventative (high dose) [22–27]. Screening will also lead to detection of more preinvasive lesions like Squamous Dysplasia and atypical adenomatous hyperplasia. Antioxidants like 2HF may be useful in these selected types of patients to prevent progression to aggressive lung cancer.

We have previously shown that the phenolic antioxidant 2-hydroxyflavanone (2HF) displays anticancer activity in RCC in a VHL-dependent manner and is associated with marked suppression of GST expression [22, 25, 27]. These studies also showed that 2HF could also inhibit the catalytic activity of GST. Some of the most potent physiological inhibitors of GSTs are GS-E, which can inhibit other enzymes GSH-linked enzymes, inhibiting efflux of GS-E can globally impair GSH-linked antioxidant and anti-apoptotic defenses utilized by cancer cells for survival [15–17]. We previously showed that GS-E transport the Ral-binding protein-1 (a 76 kDa splice variant protein referred to as RLIP76, or simply Rlip, encoded by the human *RALBP1* gene) is a high-capacity ATP-dependent transporter responsible for the bulk of GS-E removal. An existential necessity of Rlip for survival of cancer cells is suggested by studies showing that Rlip deficiency strongly prevents benzo[a] pyrene induced carcinogenesis [17]. The magnitude of this cancer preventative effect was evident in recently reported studies showing that Rlip haploinsufficiency is sufficient to prevent spontaneous carcinogenesis in *TP53* null mice [28]. Depleting Rlip by antisense or siRNA, or inhibition by anti-Rlip antibodies causes regression, not simply a growth delay, of syngeneic melanoma, and allogeneic xenografts of human neuroblastoma, and lung as well as kidney, prostate, pancreas, and colon cancer [29]. Thus, Rlip targeting should also have a therapeutic role in established malignancy.

We studied the effects of 2HF in lung cancer cell lines and found that 2HF displays strong anticancer activity in both small cell and non-small cell histologies of lung cancer associated and present evidence of direct interaction of 2HF with Rlip.

## RESULTS

### Rlip is expressed human lung cancer

The expression of the Rlip analyzed showed remarkable differences amongst the human adenocarcinoma of lung tissue sections and adjacent normal tissue. Using immunohistochemistry (IHC), tissues affected with adenocarcinoma showed significantly strong Rlip expression (Figure 1A) in cancerous tissues. On the contrary, adjacent normal tissue showed basal Rlip expression. Quantification of Rlip expression (Figure 1B) in tissues using image pro, reveals a significant difference (*p* = 0.0386) in staining intensity of Rlip between cancerous tissue and the adjacent normal tissue. Thus, higher Rlip expression may be responsible for drug resistance in lung cancer patients.

**Figure 1:** Immunohistochemistry analysis of Rlip protein expression in human adenocarcinoma of lung tissue sections Unidentified lung cancer and adjacent normal lung tissue were analyzed by IHC using anti-Rlip antibodies and representative photomicrographs are shown (**A**). IHC quantification of Rlip expression in tissues was performed using image pro (**B**) (*n* = 8).

### 2HF inhibited growth and survival of lung cancer cell lines

Concentration dependent growth inhibitory effects of 2HF was also observed in the *TP53* wild-type squamous cell histology H520 and H358 NSCLC cell line, and well as in the *TP53* mutant H1417 and H1618 SCLC cell lines. The two SCLC cell lines were somewhat more sensitive to 2HF (average GI_50_ 21 μM) than the NSCLC cell lines (average GI_50_ 52 μM, *p* < 0.01) (Figure 2A). Clonogenic assays confirmed that 2HF inhibited lung cancer cell survival as shown for the H358 and H520 NSCLC cell lines (54 and 46% inhibition, respectively, *p* < 0.001). The immortalized non-malignant human lung bronchioepithelial cell line HLBEC grew significantly slower than the malignant cell lines as expected and its survival was not significantly affected by 2HF in clonogenic assays (Figure 2B). The GI_50_ of 2HF towards these lung cancer cell lines ranged from 20 to 80 μM, in a concentration range observed for many ‘generally regarded as safe’ natural compounds that are sufficiently non-toxic to achieve these concentrations *in-vivo* upon oral dosing, even in humans [23]. Importantly, 2HF inhibited the growth of ALK (anaplastic lymphoma kinase) gene-rearranged H3122 and H2228 adenocarcinoma NSCLC cell lines. This is significant because ALK rearranged adenocarcinomas are resistant to the commonly used EGFR kinase inhibitors. Furthermore, the H2228 cell line displays acquired resistance to ALK-inhibition, GI_50_ of 2HF being 84 ± 5 *vs* 62 ± 5 μM for H2228 and H3122, respectively (*p* < 0.01) (Figure 2C).

**Figure 2:** Anticancer activity of 2-hydroxyflavonone and effect of Rlip expression in lung cancer cell lines We examined the differential toxicity of 2HF in non-malignant human lung bronchioepithelial cells (HLBEC) compared with the H1417 and H1618 SCLC and the H358 and H520 NSCLC cell lines (**A**). The cytotoxicity of 2HF on the H358 and H520 NSCLC cell lines was further confirmed by a colony-forming assay is shown (**B**). The growth inhibitory activity of 2HF toward ALK-rearrangement harboring H3122 and H2228 cell line (**C**). The growth inhibitory effect of polyclonal rabbit-anti-human anti-Rlip IgG was determined by MTT assays on H358 or H1618 lung cancer cells treated with varying antibody concentration (0–60 μg/mL) at 72 h after addition of antibody to cells in log-phase of growth (**D**). We performed the effects of anti-RLIP76 IgG and 2HF (5 and 10 μM conc.) and their combination on the survival of H1618 (SCLC) and H358 (NSCLC) cells using MTT assay (**E**). Control antibodies were the purified IgG fraction from pre-immune serum. MTT assays were performed according to our previously published standardized methods. Anti-Rlip and pre-immune IgG fractions were purified from rabbit sera provided by Alpha Diagnostics (San Antonio, TX).

### 2HF enhanced growth effect of Rlip inhibition

We have previously shown that anti-Rlip antibodies bind to a cell surface epitope of Rlip and exert potent and specific growth-inhibitory and pro-apoptotic effects against a wide variety of human SCLC and NSCLC cell lines *in-vitro* and *in-vivo* [30]. We reasoned that 2HF would potentiate the effects of these antibodies. Using MTT assays, we confirmed that the polyclonal anti-Rlip antibodies used in present studies exhibited similar growth inhibitory effects towards SCLC and NSCLC as previously observed (Figure 2D). Sub-GI_50_ concentrations of 2HF (5 and 10 μM) inhibited growth of H1618 SCLC by 21 ± 8% and 28 ± 7%, respectively and of H358 by 14 ± 5% and 19 ± 5%, respectively. At 10 μg/ml anti-RLIP76 IgG itself inhibited growth of H1618 by 20 ± 7% and H358 by 16 ± 5%, respectively. Together, 10 μg/mL anti-RLIP76 IgG and 5 or 10 μM 2HF exerted supra-additive growth inhibition (61 ± 4% and 81 ± 6% in H1618; 46 ± 3% & 68 ± 4% in H358) (Figure 2E).

### 2HF reduced protein level and inhibited the transport activity of Rlip

We found that cellular content of Rlip protein was significantly reduced by 25 μM 2HF. At 24 h after treatment with 25 μM of 2HF, the expression of RLIP76 was reduced to approximately half. This effect was manifested similarly in the H358 NSCLC and H1618 SCLC cell line, earlier than the appearance of significant apoptosis (Figure 3A). The anthracycline chemotherapy drug doxorubicin (DOX) is a model transported substrate (allocrite) for transport by purified recombinant Rlip reconstituted into lecithin: cholesterol artificial liposomes [31]. In this assay, purified Rlip protein from NSCLC has been shown to display higher specific activity for DOX transport than that purified from SCLC cell lines [30]. To determine whether 2HF inhibited Rlip transport activity, we measured DOX transport activity of Rlip protein purified from H358 and H1618 cell lines and reconstituted into artificial liposomes. Control liposomes prepared in the absence of Rlip protein displayed no uptake of ^14^C-DOX, whereas ATP-dependent uptake was clearly evident in liposomes reconstituted with Rlip protein from SCLC or NSCLC cell lines. Specific activity of transport (nmol/min/mg protein) was greater for Rlip from NSCLC than SCLC as previously observed [30]. At 10 μg/mL, anti-Rlip IgG inhibited transport whereas pre-immune IgG did not. At 20 μM, 2HF reduced DOX transport by 22 and 25% for NSCLC and SCLC, respectively. This concentration of 2HF synergistically enhanced the transport inhibition by anti-Rlip antibodies, to 93 and 95% by Rlip from NSCLC and SCLC respectively (Figure 3B and 3C).

**Figure 3:** Effects of 2HF on expression and activity of Rlip Western-blot analyses for RLIP76 were performed on control (C) as well as 25 μM of 2HF treated (T) H358 and H1618 lung cancer cells. Aliquots of 50 μg crude membrane fraction were loaded in SDS-PAGE, transblotted, and probed with anti-Rlip IgG, and developed bands were quantified by scanning densitometry. β-actin expression was used as loading control. Depletion of RLIP76 in lung cancer cells by 2HF was comparable to the results with RLIP76-antisense (10 μg/mL conc.) mediated knockdown of RLIP76 (**A**). Effects of anti-RLIP76 IgG (10 μg/mL conc.) and 2HF (10 and 20 μM conc.) and their combination on the transport of ^14^C-DOX in purified reconstituted vesicles prepared from H1618 and H358 cells were also performed by rapid-filtration technique using 250 ng protein per 30 μL reaction mixture (**B** and **C**).

### Docking of 2HF at the DNP-SG binding site of Rlip

Rlip protein bound to the dinitrophenyl-S-glutathione (DNP-SG) affinity resin could specifically eluted by with 50 and 100 μM 2HF (Figure 4A). Specificity of elution was evident because the same major Rlip protein bands were observed in the 2HF eluate as in the DNP-SG eluate. Additionally, a marked increase in elution of Rlip protein by 2HF was observed in the presence of ATP, a finding identical to that with DNP-SG (Figure 4A). Elution pattern of eluted Rlip peptides resembles with our previous purifications, that they have been confirmed by mass to be fragments of Rlip that 38 kDA is DNP-SG ATPase (the former designation of Rlip) [32–34]. Because the concentrations of 2HF that effectively eluted Rlip by displacing DNP-SG are similar to those necessary for cytotoxicity in NSCLC cell lines, it was reasonable to conjecture that 2HF and DNP-SG shared a common binding site on Rlip. We explored this possibility by defining the DNP-SG binding site of Rlip through site-directed mutagenesis. Point mutants of Rlip were created at residues Y231, R232, S234, A264, S265, K268, I344, V345 and the allocrite-stimulated ATPase activity was determined (Table 1).

**Figure 4:** Docking of 2HF, DNPSG and ATP to RLIP76 (**A**) Binding interaction of RLIP with 2HF was demonstrated by elution of recombinant RLIP with elution buffer containing 2HF. (**B**) shows binding modes of 2HF and DNP-SG at the R232 site. (**C**) 2HF forms a hydrogen bond with Q269 and cation-π interaction with K237. (**D**) DNP-SG forms hydrogen bond/salt bridge network with R232/S234/K268/N341. (**E**) ATP also prefers binding at the ATP-binding pocket of Rlip forming 5 H-Bonds to G235, K237, S265, K268 and R272. Details are given in the Materials and Methods section.

**Table 1:** ATPase activity of Rlip and its mutants^*^

Protein	specific activity (nmol/min/mg)	
	DOX	DNP-SG
**RLIP76**	275 ± 7	220 ± 15
**M1**	145 ± 1	95 ± 11
**M2**	105 ± 20	75 ± 4
**M3**	150 ± 1	175 ± 4
**M4**	205 ± 16	60 ± 7

^*^Mutants designated as M1 through M4 were mutated at the following residues: M1 (Y231A;R232A;V233K,S234A); M2 (A264R;S265A;L267A;K268A); M3 (Q340A;N341A); M4 (I344A;V345A)

We used three-dimensional NMR structure of the human RLIP76 RhoGAP-Ral binding domain with 265 amino-acid residues (RCSB protein databank PDB ID 2 mbg [35]) as model to dock the small molecules by using our in-house developed All-Around Docking (AAD) method [36] which can predict the best docking site of a ligand, together with the induce fit docking (IFD) method that allows side-chain flexible for model refinement (Schrödinger, New York, NY). The three-dimensional structural docking model revealed that 2HF and DNP-SG can both bind to the R232 site in similar proximity (Figure 4B). 2HF may form one hydrogen bond (HB) with Q269 and cation-π interaction with K237 (Figure 4C), and DNP-SG forms HBs/salt-bridge with R232, S234, K268 and N341 (Figure 4D). The ATP molecule is also predicted to bind this site (Figure 4E), forming HB network with G235, K237, S265, K268 and R272.

### CDNB co-treatment can reduced DOX efflux and GI_50_ of 2HF

We have shown that 2HF inhibits Rlip expression, Rlip transport activity and DOX efflux in cancer cells. CDNB (1-chloro-2,4-dinitrobenzene) is an alkylating agent previously used for treatment of skin metastases of melanoma through intralesional injection [37]. It is used as a model substrate for GST, which conjugates it with GSH to form S-(2,4-dinitrophenyl)-glutathione (DNP-SG) *ex-vivo* [38, 39] and is used to measure GST activity. Furthermore, conjugation of GSH in cells with CDNB causes over 98% depletion of GSH in cancer cell lines as well as *in-vivo* lymphocytes (GSH- measurement method; sulfasalazine). GS-E are known to be highly effective competitive inhibitors of transport of other allocrites by Rlip [40]. Therefore, we conjectured that DNP-SG formed in cancer cells would increase Rlip-inhibitory activity of 2HF and synergistically potentiate its anticancer activity. Consistent with this assertion, CDNB lowered the GI_50_ of 2HF significantly (*p* < 0.05) in H358 cells (Table 2). Furthermore, the time-dependent efflux of DOX was impaired significantly by CDNB as well as 2HF. The half life of DOX removal from cells was determined 12 min, 16 min and 18 min for 1 μM DOX, 1 μM DOX+50 μM 2HF and 1 μM DOX+50 μM 2HF+20 μM CDNB, respectively (Figure 5).

**Table 2:** GI_50_ of CDNB, 2HF and 2HF in presence of CDNB on H358 lung cancer cells

H358 NSCLC	
Substrate	GI_50_ (μM)
CDNB	2.83 ± 0.148
2HF	25.44 ± 0.671
2HF in presence of 1 μM CDNB	8.25 ± 0.786

**Figure 5:** Effects of 2HF and/or CDNB on DOX efflux DOX efflux studies were performed in presence and absence of 2HF and CDNB as described in Materials and Methods section. Loss of DOX was calculated and rate constant was determine to demonstrate inhibition of DOX efflux in H358 cells.

### 2HF reduced expression of genes responsive to Rlip depletion

We have previously observed [41] that Rlip deficiency causes differential expression changes in other GSH-linked stress defense enzymes. 2HF inhibited the transport activity of Rlip and reduced its expression at the protein and mRNA level. Therefore, we determine the effects of 2HF (50 and 100 μM) on adenocarcinoma (A549-p53 WT) and squamous cells (H226-p53MUT), on expression of several key MPy mRNA (Figure 6). Based on the effects of 2HF on mercapturic acid pathway gene mRNA expression in cell lines, we identified a set of seven genes that predicted opposite survival effects in adeno and squamous carcinoma: worsened in adeno and improved in squamous. This gene set predicted survival better than p53 status.

**Figure 6:** Effect of 2HF on selected MPy gene expression Expression level of MPy genes was determined by qPCR. A549 and H226 cells grown in 100 mM tissue culture Petri dishes were treated with vehicle, 50 μM or 100 μM 2HF for 24 h. Total RNA and then cDNA was prepared from harvested cells using standard methods described in Materials and Methods section. qPCR was performed using gene-specific primers.

### 2HF inhibited NSCLC and SCLC xenografts in nude mice

H1618 and H358 lung cancer cells bearing animals with established s.c. implanted tumors (~20 mm^2^) were treated with 2HF (7 mg/kg b.w.) in corn oil by oral gavage on alternate days. At this dose, 2HF was well tolerated without any overt toxicity or weight loss (Figure 7A). The product of bi-dimensional tumor measurements revealed significant growth inhibition of H358 and H1618 cell lines (Figure 7B). Excised tumors from 2HF treated mice were visibly smaller and tumor weight was significantly lower (Figure 7C and 7D). At day 60, the tumor cross-sectional area and tumor-weight of mice bearing H1618 and H358 cells was significantly lower in 2HF treated group as compared to the vehicle only (corn-oil) treated group (H1618: area 47.4 ± 6.2 mm^2^ *vs.* 129 ± 11 mm^2^ and weight 0.71 ± 0.1 g *vs.* 2.01 ± 0.23 g, *p* < 0.001; H358: area 53.5 ± 6.8 mm^2^ *vs.* 137 ± 11 mm^2^ and weight 0.92 ± 0.12 g *vs.* 2.32 ± 0.21 g, *p* < 0.001). Euthanasia was performed at 24 h after the last dose of 2HF and steady-state 2HF levels in the serum by LC-MS were found to be 5.2 and 3.8 μM in the H1618 and H358 mice, respectively. 2HF metabolites were not measured. Taken together, these results showed that orally administered 2HF is systemically absorbed and exhibits antitumor activity against an SCLC and an NSCLC human cell line in a mouse xenograft model without overt toxicity.

**Figure 7:** Anticancer activity of 2HF towards SCLC and NSCLC Hsd: Athymic nude nu/nu mice were obtained from Harlan, Indianapolis, IN. Ten 10-weeks-old mice were divided into two groups of 5 animals (treated with corn oil (vehicle), and 2HF compound 7 mg/kg b.w.). All animals were injected with 1 × 10^6^ H1618 cells suspensions in 100 μL of PBS, subcutaneously into one flank of each mouse. Treatment was started 10 days after the implantation to see palpable tumor growth. Treatment consisted of 0.2 mg of 2HF/mice in 200 μl corn oil by oral gavage alternate day. Control groups were treated with 200 μL corn oil by oral gavage alternate day. Experimental details are given in the Materials and Methods section. Animals were examined daily for signs of tumor growth and body weights were recorded. Animal weights (**A**) and product of bi-dimensional tumor measurements (**B**), photographs of dissected tumors (**C**) and tumor weights (**D**) are shown. Control and 2HF treated lung cancer bearing nude mice tumor sections were used for histopathologic analyses. Presented are H&E stained sections, IHC analyses for Ki67 expression (marker of cellular proliferation), CD31 (angiogenesis marker), and E-cadherin (tumor suppressor) from tumors in mice of control and 2HF-treated groups. Statistical significance of difference was determined by two-tailed Student's *t* test. *p* < 0.001, 2HF-treated compared with control. Immuno-reactivity is evident as a dark brown stain, whereas non-reactive areas display only the background color. Sections were counterstained with Hematoxylin (blue). Photomicrographs at 40x magnification were acquired using Olympus DP 72 microscope. Percent staining was determined by measuring positive immuno-reactivity per unit area. Arrows represent the area for positive staining for an antigen. The intensity of antigen staining was quantified by digital image analysis using Pro Plus software. Bars represent mean + S.E. (*n* = 5); ^*^p < 0.001 compared with control (**E**). Western-blot analyses of signaling proteins in H1618 and H358 human lung cancer tumor tissue lysates in control and 2HF treated experimental groups. GAPDH was used as a loading control (**F**). The bar diagrams represent the fold change in the levels of proteins as compared to controls as determined by scanning densitometry. Dotted line represents no significant change as observed with control (**G**).

### 2HF treated tumors exhibited broad anticancer signaling effects in tumors

Immunohistochemical examination of paraffin-embedded tumor xenograft sections revealed that 2HF treatment was associated with decreased expression of the proliferation marker Ki67 and the angiogenesis marker CD31. E-Cadherin, a protein that inversely correlates with invasion and growth of many epithelial cancers, was increased (Figure 7E). Western-blot analyses of the tumor tissue lysates from 2HF treated mice revealed reduction in cell growth promoting signals such as AKT and p70S6K, proliferation signals such as CDK4 and cyclin B1. Increased apoptosis was evident from changes in BH3 domain apoptosis regulatory proteins, with the anti-apoptotic Bcl-2 being reduced and pro-apoptotic Bax being increased. Epithelial-mesenchymal transition signaling was also reduced as indicated by reduction in vimentin and fibronectin and increase in E-cadherin. Thus, we conclude that 2HF induces apoptosis, inhibits cell cycling and growth signaling by modulating the expressions of BCL2 (B-cell lymphoma 2), BAX (BCL2 Associated X, Apoptosis Regulator), CDK4 (Ser/Thr-kinase component of cyclin D), cyclin B1, PIK3CA (phosphatidylinositol-4,5-bisphosphate 3-kinase catalytic subunit alpha), AKT (Protein kinase B) and p70S6K (phosphoprotein 70 ribosomal protein S6 kinase) in lung tumor.

## DISCUSSION

In previous studies, we found that the anticancer activity of 2′-hydroxyflavanone (2HF), a citrus flavonoid, against renal carcinogenesis is associated with the inhibition of glutathione S-transferases (GSTs), the first step enzyme of the mercapturic acid pathway (MPy). Since the MPy enzymes are upregulated in lung cancer, we evaluated the anti-carcinogenic activity of 2HF in SCLC and NSCLC cell lines. We showed by immunohistochemistry that Rlip protein is present in human lung cancer and its level are increased in lung cancer cells compared with surrounding normal tissue. Inhibition of epithelial-mesenchymal transition was indicated by increased E-cadherin and reduced fibronectin and vimentin. 2HF reduced mercapturic acid pathway activity by reducing the expression as well as transport activity of the Rlip. Inhibition of doxorubicin efflux by 2HF increased its accumulation in the cells, but 2HF did not add to the transport inhibitory effect of anti-Rlip antibodies alone. Binding of Rlip to 2HF was evident from successful purification of Rlip by 2HF affinity chromatography. Consistent with increased drug accumulation, combined treatment with 1-chloro-2,4-dinitrobenzene, which is converted to a glutathione conjugate in cells, reduced the GI_50_ of 2HF by an order of magnitude. We have previously shown that Rlip is a major determinant of the inherent chemoresistance of NSCLC compared with SCLC and results of present studies showing that 2HF potentiated the apoptotic effect of anti-RLIP76 antibodies in SCLC as well as NSCLC in cell culture support our previous results. Orally administered 2HF inhibited growth of xenografts of SCLC and NSCLC cell lines in nu/nu mice. The anticancer activity of 2HF *in-vitro* was preferentially directed towards malignant cell lines and was confirmed in these *in-vivo* xenograft studies where we found excellent tolerability and lack of significant toxicity of orally administered 2HF.

Our previously published studies have consistently shown greater activity of Rlip-targeting in SCLC as compared with NSCLC [42]. Mimicking human disease, SCLC cell lines are generally more sensitive to many clinically available chemotherapy drugs (doxorubicin, vincristine, cyclophosphamide and others), than NSCLC [42–44]. Chemosensitivity of SCLC results in a rapid response, but relapse with refractory cancer occurs in the vast majority due to residual resistant populations of treatment-resistant cancer stem-cells [45]. SCLC cell lines are known to have frequent loss of p53 in SCLC [46] and p53 deficiency is known to cause promoter demethylation of cancer stem cell genes [47]. Taken together with our recent studies showing that Rlip depletion in *Tp53*^−/−^ mice nearly completely prevents the hypomethylation of the promoters of many stem cell genes [28], suggest that 2HF could overcome cancer stem-cell mediated therapy resistance of p53-mutated SCLC. Treatment resistant stem cell have also been demonstrated in lung SqCA [48], thus effects of 2HF on cancer stem-cell gene could translate into clinical activity in this subtype of NSCLC. Consistent with our previous studies in multiple histologies of cancer [22, 23, 30, 49–52], we found that Rlip targeting exerts anticancer effects regardless of the presence of normal p53. This is relevant to lung AdCA, nearly half of which lack genetic lesions in p53.

We have previously shown that 2HF can inhibit expression as well as the catalytic activity of GST [26, 53], the first committed step of the MPy. Present studies show that 2HF also inhibits both expression and transport activity of Rlip, the next and rate-limiting step of the Mpy. Synergy between 2HF and anti-Rlip antibodies in their anti-cancer activities supports the importance of Rlip and the MPy in the mechanisms of action of 2HF. Regulation of redox-regulating genes by Rlip, and the regulation of Rlip by transcription factors involved in oxidative stress response suggests a possible mechanism for the anticancer activity of 2HF because Rlip inhibition would have a broad impact on the generation of pro-apoptotic oxidative metabolites contributing to anticancer activity of 2HF [54–56].

Similar to several other plant phenols [57], the anticancer activity of 2HF seem to be associated with pleiotropic effects on multiple cancer signaling pathways that regulate cell growth and proliferation, epithelial-mesenchymal transition (EMT), apoptosis, and angiogenesis. The cellular concentration of E-cadherin was increased by 2HF exposure, which was paralleled by a decrease in vimentin and fibronectin, paradigmatic for inhibition of EMT [58]. E-cadherin is considered a suppressor of invasion and growth of many epithelial cancers because of its role in inhibition of EMT and promoting normal epithelial phenotype [59]. EMT is intimately linked to a higher availability of growth factors, such as insulin like growth factor (IGF) [60], membrane metalloproteases (MMPs) [61], and an increase in vascularity [62]. This is paralleled by a repression of certain transcription factors [63] and cytoskeletal proteins [64] and finally by the development of matrix independent growth and corresponding tumor cell progression and metastasis formation [65]. In correlative studies the occurrence of EMT has been associated with a more aggressive phenotype, the resistance to chemotherapy and biologic agents and a poor prognosis [66]. In addition, we demonstrated a striking reduction of fibronectin. Fibronectin, which is assembled in the extracellular matrix, is involved in several biologic functions, including in cell adhesion, growth, migration, and differentiation. It is increased in NSCLC subtypes and has been linked to cross pathway activation and radiation-resistance [67]. Since EMT signaling plays a key role in maintenance of cancer stem cells, our findings predict that 2HF can be useful in overcoming the treatment resistance conferred by the persistence of highly resistant cancer stem-cells.

Bax and Bcl-2 are both key members of the Bcl-2 family of proteins that are functionally linked with mitochondria and intimately involved in the late signaling phase of intrinsic apoptotic cell death [68]. Increased Bcl-2 and reduced Bax have been linked to the malignant phenotype, and correlated with survival advantage [69]; in normal bronchioepithelial cells, the opposite is true. Early studies of the Bcl-2 family have suggested that p53 loss up-regulates Bcl-2 and is associated with the loss of Bax transactivation and Bax has been shown to regulate apoptosis in lung cancer patients [70]. Chemotherapy resistance of p53-mutated tumors has been attributed to the loss of transactivation of anti-apoptotic Bax and more recently increased levels of Bcl-2 have been linked to a poor outcome in SCLC [71]. Both cell lines we investigated carry genetically altered p53, H358 having a homozygous deletion of the p53 gene [72] and H1618 having a p53 exon 248 mutation [73]. When compared to untreated animals, 2HF demonstrate the down-regulation of anti-apoptotic Bcl-2 which is paralleled by an increased in pro-apoptotic Bax.

The PI3K/Akt/mTOR pathway governs the growth of cancer cells and has been the subject of intense interest in cancer therapy. Phosphorylated Akt has been described to be a negative prognosticator in lung cancer [74] and an increased level can be observed early in lung cancer carcinogenesis [75] and in therapeutic resistance [76–78]. In addition, activation of the pP70S6 Kinase is as an important distal event in the intracellular signal transduction of several growth factor pathways, including the insulin like growth factor pathway. It should be noted that Rlip targeting alone blocks the same signaling pathway in other cancers [79], and perhaps more remarkably, that this pathway is actually activated by Rlip depletion in non-malignant cells [80]. The fundamentally opposite effect of Rlip on this pathway may underlie low toxicity towards non-malignant cells. Additionally, greater expression of Rlip in cancer compared with normal tissue suggest a greater dependence of cancer cells on Rlip and could also contribute to improved selectivity towards lung cancer cells.

In addition to inhibiting the PIK3CA/AKT/p70S6K pathway that promotes the growth of cells, we found the cell cycling and proliferation were also affected, as evidenced by reduction in CCNB1 and CDK4 protein. Both proteins are intimately related to cell cycle progression and an increase in their levels has been linked to an adverse prognosis in lung cancer [81, 82]. Cyclin B1 in conjunction with cdc2 (Cdk1) forms a complex called the ‘mitotic promoting factor’ (MPF), which crucial for G2/M transition [83]. We and others have previously shown that Rlip also interacts directly with cdc2 (CDK1) [84]. Reductions of cyclin B-CDK1 complex levels are related to cell cycle arrest at G2 and finally DNA fragmentation [85]. It is felt that this is one of the major molecular processes accounting for the anti-neoplastic effect of p53 associated cisplatin activity. Intriguingly, this mechanism is different from the DOX-induced apoptosis in SqCA, which is associated with heightened levels of cyclin B1 in the process of mitotic catastrophe. In addition to its value as a negative prognostic marker, CDK4 has been more recently targeted in other malignancies with clinical success [82, 85].

## MATERIALS AND METHODS

### Reagents

MTT and 2HF were obtained from sigma (St Louis, MO). CD31, Ki67, cyclin B1, CDK4, cleaved PARP, vimentin, Akt, pAKT (S^473^), fibronectin, Bax, Bcl2, P70S6K, pP70S6K (S^S240–244^), PI3K, and E-cadherin antibodies were purchased from Santa Cruz Biotechnology (Columbus, OH) and Cell Signaling Technologies (Danvers, MA). ^14^C-DOX (doxorubicin: specific activity 58 mCi/mmol) was purchased from NEN Life Sciences (Boston, MA). Matrigel was procured from BD Biosciences (San Jose, CA). TUNEL fluorescence and avidin/biotin complex (ABC) detection kits were purchased from Promega (Madison, WI) and Vector (Burlingame, CA), respectively. Ninety-six well nitrocellulose membrane plates (pore size 0.45 μm) used in transport studies were purchased from the Millipore Co. (Bedford, MA). The source of anti-RLIP76 antibodies and DNP-SG were the same as previously described [32]. All other reagents were of analytical grade.

### Cell lines and cultures

Human SCLC (H1417 and H1618) and NSCLC (H358 and H520) were purchased from ATCC, Manassas, VA. Human lung bronchoepithelial (HLBE) cells were a generous gift from Dr. John D. Minna, University of Texas Southwestern Medical Center, Dallas, TX. All cells were cultured at 37°C in a humidified atmosphere of 5% CO_2_ in RPMI-1640 medium supplemented with 10% FBS and 1% P/S solution except HLBEC, which grow in K-SFM. The cells were immediately expanded and frozen after being obtained from ATCC and restarted every 3 to 4 months from a frozen vial of the same batch of cells and no additional authentication was done on these cells. All cells lines were free of Mycoplasma infection tested by PCR.

### RLIP76 expression in lung cancer

Immunohistochemistry of human adenocarcinoma of lung tissue sections was performed on 5-μm thick serial sections prepared from formalin-fixed paraffin-embedded tissue, using monoclonal mouse anti-RalBP1 IgG from Santa Cruz (sc-48337). Tissue sections were de-paraffinized in xylene and rehydrated in graded alcohol. This was followed by antigen retrieval (5 mL antigen un-masking reagent + 1 mL EDTA (0.5 M) in 500 mL water) by steaming. The slides were placed in incubation chamber and blocked with 1% human serum albumin at room temperature for 1 h. The anti-Ralbp1 IgG (from Santa Cruz) was added (1:25 dilution) and incubated at 4^°^C overnight and the slides were washed in 1x PBS+ 0.2% Triton X-100 by incubating for 5 min at shaker with gentle shaking. Slides were stained using the ABC universal kit (Vector) following manufactures instructions, counterstained with hematoxylin, and mounted. All images were acquired at a fixed distance, using the same channel settings (exposure times, laser intensities) using Olympus BH2 microscope at Anatomical Pathology Lab at the City of Hope. All human subject studies were approved by the COH (IRB#11175) and carried out in accordance with their guidelines.

### Drug sensitivity (MTT) assay

Cell density measurements were performed using a hemacytometer to count intact cells resistant to staining with trypan blue. Approximately 20,000 cells were plated into each well of 96-well flat-bottomed micro-titer plates. After 12 h incubation at 37°C, medium containing either pre-immune IgG or anti-RLIP76 IgG (ranging 0–60 μg/mL final conc.) were added to cells followed by incubation for 24 h, then 2HF (ranging 0–200 μM) were added to cells. After 48 h incubation, 20 μL of 5 mg/mL MTT were introduced to each well and incubated for 2 h of exposure. The plates were centrifuged and the medium was decanted. Cells were dissolved in 100 μL DMSO with gentle shaking for 2 h at room temperature, followed by measurement of OD_570_ [41]. Eight replicate wells in each of three separate measurements. For GI_50_ determination of CDNB and 2HF ±CDNB in H358 cells, approximately 5,000 cells were plated as above in 96 well plate. After 12 h cells were treated with 0–15 μM CDNB or 0–150 μM 2HF and 1 μM CDNB+0–150 μM 2HF. After 48 h MTT assay was performed as described above.

### Colony formation assay

Cell survival was evaluated using a standard colony-forming assay. 1 × 10^5^ cells / mL were incubated with 2HF (50 μM) for 24 h and aliquots of 50 and 100 μL were added to 60 mm size Petri dishes containing 4 mL culture medium. After 10 days, adherent colonies were stained with 0.5% methylene blue for 30 min and counted using Innotech Alpha Imager HP [86].

### DOX efflux study

1.5 × 10^5^ H358 cells were plated in chamber slides. After overnight incubation at 37°C in a 5% CO_2_ atmosphere, cells were exposed with 1 μM DOX for 16 h followed by treatment with vehicle, 20 μM 2HF or 20 μM 2HF+20 μM CDNB for 4 h. Cells were gently washed, added 2 ml of PBS and placed the chamber slides on a magnetic stirrer with magnetic bar in each chamber. Every 2 min for 30 min, 50 μL aliquot of the effluent from each well was taken and placed in a black 96 well flat bottom plate. Fluorescence was measured by using of infinite M1000Pro (Tecan) with 500/550 nm for excitation and emission wavelength setting.

### Docking studies

The predicting binding modes of 2HF, DNP-SG and ATP molecule in complex with RLIP76 were calculated by using our in-house developed All-Around Docking method [36] and the Glide XP docking tools of Schrödinger suite of software [87]. The human RLIP76 RhoGAP-Ral domain three-dimensional NMR structure were obtained from protein data bank with 265 amino-acid residues (RCSB protein databank PDB ID 2 mbg [35]). First, we performed All-Around Docking for small molecules 2HF, DNP-SG and ATP to search the human RLIP76 protein three-dimensional surface for the best docking site(s). Thereafter with the induced fit docking, which allows side-chain of the pocket residues to be flexible for more accurate computation of the binding modes, the complex models were refined with docking score as −6.7 for DNP-SG, −5.1 for 2HF and −9.8 for ATP.

### Effect of 2HF on RLIP76 expression

H358 and H1618 cells were treated with 25 μM of 2HF for 24 h at 37°C followed by washing with PBS, re-suspended in the medium, and allowed to recover for 2 h. Cells were solubilized in lysis buffer and centrifuged at 105,000 × g for 1 h at 4°C, and the supernatant was collected. 50 μg of proteins were subjected to SDS-PAGE followed by Western-blot analyses using anti-RLIP76 IgG.

### Quantitative (real-time) PCR

A panel of transcripts encoding enzymes involved in 4-HNE metabolism and in general antioxidant defense was quantitated by PCR. Total RNA was isolated from A549 and H226 cells treated with 50 or 100 μM 2HF for 24 h using TRIZOL reagent. DNase-treated total RNA was used for first DNA strand synthesis (superscript II, Invitrogen). Real-time quantitative PCR (QPCR) amplification reactions were performed with the SYBR Green qPCR kit (Roche) using 5 μL of cDNA and 0.3 μM gene-specific primers.

### Purification of RLIP76

DNPSG-affinity purification of RLIP76 from SCLC (H1417 & H1618) and NSCLC (H358 & H520) cells was carried out as described previously [50]. Purifications were monitored by measuring transport activity. To demonstrate 2HF competitively bind to RLIP, we eluted recombinant RLIP with elution buffers containing 2HF with or without ATP. Eluted protein was separated on NuPAGE 4–12% Bis-Tris Protein Gels (Invitrogen) followed by transfer on nitro cellulose membrane. Purified protein was identified using anti Rlip antibody. Compositions of elution buffer used in purification are as follows: Elution buffer1: 10 mM ATP+ 10 mM MgCl_2_+ 0.025% C_12_E_9_+ 0.2 mM DNP-SG in Lysis buffer (Original) [32–34]; Elution buffer2: Original lysis buffer with no ATP, No DNP-SG; Elution buffer3: 1 mM ATP+ 50 μM of 2HF (no DNP-SG); Elution buffer4: 1 mM ATP+ 100 μM of 2HF (no DNP-SG); Elution buffer5: no ATP + 100 μM 2HF (no DNP-SG)).

### Reconstitution of purified Rlip into artificial liposomes

Purified Rlip from lung cancer cells was dialyzed against reconstitution buffer (10 mM Tris-HCl, pH 7.4, 4 mM MgCl_2_, 1 mM EGTA, 100 mM KCl, 40 mM sucrose, 2.8 mM β-mercaptoethanol, 0.05 mM BHT, and 0.025% polidocanol), and reconstituted into artificial asolectin-cholesterol liposomes. An aqueous emulsion of soybean asolectin (40 mg/mL) and cholesterol (10 mg/mL) was prepared in the reconstitution buffer by sonication, from which a 100 μL aliquot was added to dialyzed purified RLIP76 protein to achieve a final concentration of 40 μg/mL. After sonication of the resulting mixture for 30 s at 50 W, 200 mg of SM-2 Bio-beads pre-equilibrated with reconstitution buffer (without polidocanol) were added to initiate vesiculation, and after 4 h incubation at 4°C, SM-2 beads were removed by centrifugation at 3000 × g and the vesicles (proteoliposomes) were collected. Control-liposomes were prepared using an equal amount of crude protein from *E. coli* not expressing Rlip [32]. The size of reconstituted vesicles was examined by electron microscopy and intra-vesicular volume was estimated by ^14^C-inulin trapping [32].

### Transport studies in Rlip-proteoliposomes

Transport studies of ^14^C-DOX in reconstituted vesicles were performed by rapid-filtration technique as described by us using 250 ng protein per 30 μL reaction mixture. ATP-dependent uptake of ^14^C-DOX (specific activity 8.6 × 10^4^ cpm/nmol, use 3.6 μM final concentration) was determined by subtracting the radioactivity (cpm) of the control without ATP from that of the experimental containing ATP, and the transport of DOX was calculated in terms of nmol/min/mg protein. Liposomes prepared without addition of Rlip were used for controls. Each determination was performed in triplicate [32].

### Transport inhibition by 2HF and anti-Rlip IgG

Purified reconstituted liposomes (250 ng protein/30 μL reaction mixture) were incubated separately with either 2HF (0–50 μM final concentration) or anti-Rlip IgG (0–60 μg/ml final concentration) or both, for 30 min at room temperature. In one of the controls, IgG was excluded while the other control was treated with an equal amount of pre-immune IgG. After incubation, the ATP-dependent transport of ^14^C-DOX was measured by using a 96 well-plate filtration manifold to separate the extra-vesicular drug from that taken up by the vesicles. Uptake was measured in Rlip-proteoliposomes and control liposomes, in absence or presence of 2HF, anti-Rlip IgG and 4 mM ATP at a fixed time point of 5 min, at 37°C.

### *In vivo* xenograft studies

Hsd: Athymic nude *nu/nu* mice were obtained from Harlan, Indianapolis, IN, and were acclimated for a week before beginning the experiment. All animal experiments were carried out in accordance with a protocol approved by the Institutional Animal Care and Use Committee. Ten 10-weeks-old mice were divided into two groups of 5 animals (treated with vehicle only i.e. corn oil, and 2HF 7 mg/kg b.w.). All 10 animals were injected with 1 × 10^6^ H1618-SCLC suspensions in 100 μL of PBS, subcutaneously into one flank of each mouse. At the same time, animals were randomized into treatment groups. Treatment was started 10 days after the H1618 cells implantation when tumors are ~20 mm^2^ in diameter (palpable tumor growth). Treatment consisted of 7 mg of 2HF/kg b.w., in 200 μL corn oil by oral gavage alternate day. Control groups were treated with corn oil only. Similar protocol was followed for H358 NSCLC xenografts studies. Animals were examined daily for signs of tumor growth. Tumors were measured in two dimensions using calipers and body weights were recorded. Each mouse in every group was monitored on alternate days for signs of distress and areas of swelling or redness. Photographs of animals were taken at day 1, day 10, day 20, day 30, and day 60 after subcutaneous injection, are shown for all groups. Photographs of tumors were also taken at day 60.

### Assessment of angiogenesis, proliferation, and apoptosis

Lung tumors (control as well as 2HF treated) were harvested from mice bearing tumors and used for histopathologic analyses. Tumor samples fixed in buffered formalin for 12 h were processed conventionally for paraffin-embedded tumor sections (5 μm thick). Hematoxylin and Eosin (H&E) staining was performed on paraffin-embedded tumor sections. Histopathologic analyses with anti-E cadherin, anti-CD31, and anti-Ki67 IgG, were also performed, using Universal ABC detection kit (Vector). Immuno-reactivity is evident as a dark brown stain, whereas non-reactive areas display only the background color. Sections were counterstained with Hematoxylin (blue). Photomicrographs at 40x magnification were acquired using Olympus DP 72 microscope.

### Analysis of cancer-signaling by western blot

The effect of 2HF treatment on signaling proteins in tumors was determined using 28,000 × g supernatant fraction of a 10% homogenate. For Western blotting, ~ 50 μg protein loaded per lane was subjected to SDS-PAGE and transferred onto the nitrocellulose membrane. Horseradish peroxidase (HRP)-conjugated anti-mouse and anti-rabbit secondary antibodies and primary antibodies towards Akt, pAKT (S^473^), PARP, vimentin, E-cadherin, Fibronectin, Bcl2, Bax, CDK4, Cyclin B1, P70S6K, pP70S6K (S^240–244^) and GAPDH were purchased from Santa Cruz Biotechnology, Inc. Detection was using chemiluminescence ECL kit (Amersham Life Sciences). GAPDH was used as loading control and representative results from one of several experiments are shown.

### Statistical analyses

All data were evaluated with a two-tailed unpaired student's *t* test and are expressed as the mean ± SD. The statistical significance of differences between control and treatment groups was determined by ANOVA followed by multiple comparison tests. Changes in tumor size and body weight during the course of the experiments were visualized by scatter plot. Differences were considered statistically significant when the *p* value was less than 0.05.

## CONCLUSIONS

Flavonoids are compounds ubiquitously present in many food sources [88]. These naturally appearing compounds have been linked to multiple biologic functions, such as anti-proliferative, pro-apoptotic, anti-inflammatory, anti-invasive and anti-angiogenic effects [26]. Present studies demonstrate that this naturally abundant, orally bioavailable and nontoxic compound exhibits tumor growth inhibitory activity SCLC and NSCLC activity by inhibiting cancer signaling and MPy, making it an attractive candidate in therapy and prevention of lung cancer.
